# Quantification of “Cold-Hot” Medicinal Properties of Chinese Medicines Based on Primary Metabolites and Fisher's Analysis

This article has been retracted.

**DOI:** 10.1155/2022/5790893

**Published:** 2022-01-22

**Authors:** Xian-rui Wang, Ting-ting Cao, Xue-mei Tian, Hui Wang, Yun Wang

**Affiliations:** Information Engineering Research Center for Traditional Chinese Medicines, Beijing University of Chinese Medicine, Beijing 102488, China

## Abstract

**Background:**

Chinese medicinal properties (CMP) are an important part of the basic theory of traditional Chinese medicines (TCMs). Quantitative research on the properties of TCMs is of great significance to deepen the understanding and application of the theory of drug properties and promoting the modernization of TCMs. However, these studies are limited to strong subjectivity or distinguish different drug properties based on certain indicators since CMP studies are diverse.

**Objective:**

To realize quantitative comparison of same medicinal properties of different Chinese medicines.

**Method:**

To solve the above problem, we proposed and explored quantification of Chinese medicinal properties (QMP) and the quantification value of medicinal properties “*R*”. The correlation between primary metabolites and “cold-hot” medicinal properties was explored on the premise of material basis of Chinese herbal medicines and Fisher's analysis. Based on indicators related to “cold-hot” medicinal properties, we utilized quantitative values “*R*” to characterize the strength or weakness of “cold-hot” medicinal properties.

**Results:**

According to QMP, the same medicinal properties were quantified and compared by quantification value of medicinal properties that expressed by alphabet “*R*”. The general theoretical formula of “*R*” deduced is *R* = (‖*l*‖ × cos *θ*)/‖*L*‖ = ∑_*i*=1_^*n*^*j*_*i*_*p*_*i*_/∑_*i*=1_^*n*^*p*_*i*_^2^, in which *n* ≥ 1. In the light of formula of “*R*” and indicators related to “cold-hot” medicinal properties, we got “*R*” value of “cold-cool” and “warm-hot” medicinal properties. “*R*” values of “cold-cool” medicinal properties of Phellodendri chinensis cortex, Coptidis rhizoma, and Menthae haplocalycis herba were 0.63, 1.00, and 0.49, respectively. The result showed that Coptidis rhizoma is the most “cold-cool”, followed by Phellodendri chinensis cortex, with Menthae haplocalycis herba is the weakest in the three Chinese medicines, consistent with cognition of TCM theory.

**Conclusion:**

QMP has certain guiding significance for the quantification of “cold and hot” drug properties. “*R*” is feasible to realize the quantitative comparison of the same drug properties of different traditional Chinese medicine, which is helpful to promote process of modern Chinese medicine construction.

## 1. Introduction

The theory of medicinal properties is an important part of basic theory of traditional Chinese medicines (TCMs), which is one of the significant guidelines to guide clinical use of TCMs [1]. The theory of medicinal properties mainly includes four natures, five flavors, channel tropism, toxicity, and ascending-descending-floating-sinking [2]. The four natures refer to four properties of TCMs that are cold, hot, warm, and cool [3], which can also be mainly classified into two categories: one is hot-warm and the other is cold-cool. The five flavors contain five basic tastes that are pungent, sweet, sour, bitter, and salty [4]. Four natures and five flavors are core of theory of medicinal properties of Chinese medicines. In particular, the study of four natures of Chinese medicines was highly sought after by researchers.

Four natures of Chinese medicines that were summarized in long-term medical practice have characteristics of abstractness, ambiguity, subjectivity, etc. [5]. Because of above characteristics, it is difficult to carry out quantitative analysis of “cold-hot” medicinal properties, which is one of the significant difficulties that impede the modernization of TCM. Quantitative analysis of “cold-hot” medicinal properties is to quantify the abstract concepts of Chinese medicinal properties “four qi” to compare the strength or weakness of “hot” or “cold” medicinal properties. Quantification of Chinese medicinal properties (CMP) that contains quantitative analysis of “cold-hot” medicinal properties is becoming a common trend in the research of TCMs [6]. The outline of strategic plan for development of TCMs had stressed that the scientific research on drug properties of TCMs should be strengthened through current scientific and technological methods. The realization of quantification of medicinal properties can strengthen people's understanding for theory of TCMs and enhance the persuasion of TCMs, which is more conducive to the modernization of TCM. To this end, relevant scholars carried out a series of exploratory research. According to Fu et al., the higher the molecular energy state and the lower the average molecular weight, the greater the correlation with the hot-warm properties of TCMs; on the other hand, the lower the molecular energy state, the greater the correlation with the cold-cool properties of TCMs [7]. Wei et al. have proposed a novel method of multisolvent similarity measure to distinguish cold-cool and hot-warm medicinal properties [8]. In addition, a research method of expert assessment has been established to quantify “cold-hot” properties of TCMs and so on [9–11].

Recently, it has become an important and urgent task for modern scientific research to identify and explain the theory of TCMs which have been applied in China for more than 4000 years. Due to the little contribution to the understanding of traditional Chinese medicine theory, the action mechanism of drugs with cold and heat characteristics is not clear. In previous quantitative study of “cold-hot” medicinal properties, however, there are some limitations in above quantitative study of “cold-hot” medicinal properties [6, 8]. For example, in the process of quantification of “cold-hot” medicinal properties, researchers adopted the subjective approach of evaluation and numerical size assignment of medicinal properties. Subjectivity is too strong to quantify medicinal properties objectively and scientifically. Moreover, most research only discriminated “cold-hot” medicinal properties based on certain indicators, rather than comparing the strong or weakness of medicinal properties [7, 10, 11]. CMP play a vital role in theoretical research and clinical practice. However, the traditional CMP system is subjective, qualitative, fixed, inconsistent, and obscured [2, 5]. Additionally, we are still short of an objective and scientific method that could realize the quantitative comparison of “cold-hot” medicinal properties of Chinese medicines. Nowadays, quantifying CMP research achieved a notable progress. We presented and analyzed quantification of Chinese medicinal properties (QMP) and the quantification value of Chinese medicinal properties “R”. From the perspective that the medicinal properties of TCMs are related to their material basis, we explored the correlation between primary metabolites and “cold-hot” medicinal properties. Further, based on indicators related to “cold-hot” medicinal properties, we utilized quantitative values “*R*” to characterize the strength or weakness of “cold-hot” medicinal properties and to realize quantitative comparison of the same “cold-hot” properties of different Chinese medicines.

## 2. Methods

### 2.1. Quantification of Medicinal Properties and Basic Rationale

#### 2.1.1. Quantification of Chinese Medicinal Properties

In this paper, we came up with a new concept—QMP. QMP proposed in this article referred to quantitative comparison of same medicinal properties of different Chinese medicines through quantification value of Chinese medicinal properties “R”, which was based on vector representation of medicinal properties and operation rules of vector and linear algebra.

#### 2.1.2. Based Rationale of Quantitative Analysis for Medicinal Properties of Chinese Medicines

In this section, we introduced the basic rationale of quantitative analysis for medicinal properties of Chinese medicines and the quantification value of Chinese medicinal properties “R”.

As shown in Figure 1, vectors *e*_1_ and *e*_2_ represent the medicinal properties of reference drug and test drug, respectively, where *θ* is the angle between the two vectors. The codirectional ray where vector *e*_1_ is located was taken as the evaluation axis of medicinal properties (EAMP). At the same time, the modulus of vector *e*_1_ was taken as the metrical unit of drug properties, with the metrical unit is expressed by “*a*”. Then, through the modulus of vector *e*_2_ and cosine value of angle *θ* to calculate vertical projection of vector *e*_2_ on EAMP, the vertical projection of vector *e*_2_ was denoted by “*b*”. On the basis of above information, we define “*b*/*a*” as the quantification value of medicinal properties of traditional Chinese medicines, which was indicated by the alphabet “*R*”. According to the rule of vectors [12], “*R*” can be strictly defined as follows:

(1) $$\begin{array}{c} R=\frac{b}{a},a=\left|e_{1}\right|,b=\left|e_{2}\right|\times \cos\theta ,\text{so }R=\frac{\left|e_{2}\right|\times \cos\theta }{\left|e1\right|}. \end{array}$$

The modulus of vector *e*_1_ was denoted as ∣*e*_1_∣; at the same time, the modulus of vector *e*_2_ was denoted as |*e*_2_|.

In addition, because the module of a vector and cos *θ* is a real number that has only size, so “*R*” is real number with no units.

There was another case where there was no clear reference drug. As shown in Figure 2, vectors *e*_1_ and *e*_2_ represented the medicinal properties of test drug *A* and test drug *B*, respectively, with vector *e*_3_ was the summation vector of *e*_1_ and *e*_2_. The codirectional ray where vector *e*_3_ located was taken as the evaluation axis of medicinal properties (EAMP); meanwhile, the vertical projections of vectors *e*_1_ and *e*_2_ on EAMP were denoted as “*b*” and “*a*”, respectively. In addition, the modulus of vector *e*_3_ was taken as a metrical unit of drug properties that was expressed by “*c*”. In the same way, we defined “*b*/*c*” and “*a*/*c*” as the quantification values of medicinal properties of test drug “*A*” and that of test drug “*B*”, respectively. Suppose that the angle between *e*_1_ and *e*_3_ is *θ*_1_, with the angle between *e*_2_ and *e*_3_ is *θ*_2_, and the moduli of vectors *e*_1_, *e*_2_, and *e*_3_ were denoted as |*e*_1_|, |*e*_2_|, and |*e*_3_|. In accordance with the rule of vectors, we can obtain that

(2) $$\begin{array}{c} e_{3}=e_{1}+e_{2},c=\left|e_{3}\right|,b=\left|e_{1}\right|\times \cos\theta_{1},a=\left|e_{2}\right|\times \cos\theta_{2},\\ R_{A}=\frac{b}{c}=\frac{\left(\left|e_{1}\right|\times \cos\theta_{1}\right)}{\left|e_{3}\right|},\\ R_{B}=\frac{a}{c}=\frac{\left(\left|e_{2}\right|\times \cos\theta_{2}\right)}{\left|e_{3}\right|}, \end{array}$$

where *R*_*A*_ and *R*_*B*_ represented the quantification values of medicinal properties of test drug “*A*” and that of test drug “*B*”, respectively.

On the basis of the above fundamentals, the quantification value of Chinese medicinal properties “*R*” was defined to realize the quantitative comparison of same medicinal properties of different traditional Chinese medicines, which can avoid the influence of subjective factors such as evaluation of experts and weight assignment of drug properties to some extent. However, a key problem to solve was how to use vectors to represent the same medicinal properties of different Chinese medicines. In the following chapters, we analyzed the question of making use of vectors to denote Chinese medicinal properties.

### 2.2. Vector Representation of Medicinal Properties

The completion of quantification of medicinal properties was on the basis of its basic rationale, but the vector representation of medicinal properties was the premise of quantification of drug properties. There are two important factors that use vectors to represent Chinese medicinal properties. One is characterization indexes of medicinal properties, and the other is coordinate representation of vector.

#### 2.2.1. Characterization Indexes of Chinese Medicinal Properties

Characterization indicator of drug properties is an “attribute index” to measure medicinal properties. Based on some “attribute index”, different drug properties of traditional Chinese medicines can be distinguished. In addition, quantifiable attribute indicators that are related to the nature of TCMs could provide a basis for quantitative comparison of medicinal properties.

More and more scientific technologies such as spectroscopy technology [13–15], high-throughput technology [16, 17], data mining [18, 19], and big data [20, 21] have been widely used in macroanalysis and microanalysis of TCMs, which provide us with a great deal of information. As far as quantitative comparison of drug properties is concerned, it is vital to select suitable characterization indexes of medicinal properties from numerous information. Therefore, when selecting the suitable characterization indicators, we should analyze the properties of characterization indexes and the connection of drug properties and indicators according to specific situation, rather than haphazard selection. The selection of characterization indicators of medicinal properties should pay attention to the following aspects:

1. There is a direct or potential connection between characterization indicators and medicinal properties
2. Characterization indicators of medicinal properties should be able to obtain corresponding indicator values rather than only described qualitatively
3. The number of characterization indicators is not less than one
4. Characterization indicators can reflect in different herbal medicines

#### 2.2.2. Coordinate Representation of Vectors

The coordinate representation of vectors is another mathematical representation of vector, which connects mathematics with vectors [22].

Supposing in the *N*-dimensional space defined as *V*, *ξ*_1_, *ξ*_2_, *ξ*_3_, ⋯, *ξ*_*n*−2_, *ξ*_*n*−1_, *ξ*_*n*_ ∈ *V*, in which *ξ*_1~*n*_ are the unit vectors with different directions;

(3) $$\begin{array}{c} \left|\xi_{1}\right|=\left|\xi_{2}\right|=\left|\xi_{3}\right|=\cdots =\left|\xi_{n-1}\right|=\left|\xi_{n}\right|=1. \end{array}$$

If $\overset{⟶}{\lambda }\subseteq V$ and $\overset{⟶}{OA}=\overset{⟶}{\lambda }$, based on the rule of summation of vectors, we can obtain the following:

(4) $$\begin{array}{c} \overset{⟶}{\lambda }=a_{1}\cdot \xi_{1}+a_{2}\cdot \xi_{2}+a_{3}\cdot \xi_{3}+\cdots +a_{n-1}\cdot \xi_{n-1}+a_{n}\cdot \xi_{n},\\ \overset{⟶}{OA}=a_{1}\cdot \xi_{1}+a_{2}\cdot \xi_{2}+a_{3}\cdot \xi_{3}+\cdots +a_{n-1}\cdot \xi_{n-1}+a_{n}\cdot \xi_{n-1}, \end{array}$$

in which *ξ*_1_, *ξ*_2_, *ξ*_3_, ⋯, *ξ*_*n*−2_, *ξ*_*n*−1_, *ξ*_*n*_ are the unit vectors fixed in *V* and point “*O*” is the origin of coordinates;

(5) $$\begin{array}{c} \overset{⟶}{OA}=\overset{⟶}{\lambda }=\left(a_{1},a_{2},a_{3},\cdots ,a_{n-1},a_{n}\right). \end{array}$$

Since the unit vectors are fixed in *V*, for any vector in *V*, there is only one set of ordered sequence (*a*_1_, *a*_2_, *a*_3,_ ⋯ , *a*_*n*−1_, *a*_*n*_) to make $\overset{⟶}{OA}=a_{1}\cdot \xi_{1}+a_{2}\cdot \xi_{2}+a_{3}\cdot \xi_{3}+\cdots +a_{n-1}\cdot \xi_{n-1}+a_{n}\cdot \xi_{n}$ set up. Then, the set of ordered sequence (*a*_1_, *a*_2_, *a*_3,_ ⋯ , *a*_*n*−1_, *a*_*n*_) is recorded as the coordinates of $\overset{⟶}{OA}$, in which the sequence is the coordinate of point “*A*”.

On the basis of the above analysis, if there are two points “*M*” and “*N*” in *V*:

(6) $$\begin{array}{c} M=\left(m_{1},m_{2},m_{3},\cdots ,m_{n-1},m_{n}\right),\\ N=\left(n_{1},n_{2},n_{3},\cdots ,n_{n-1},n_{n}\right),\\ \xi_{1},\xi_{2},\xi_{3},\cdots ,\xi_{n-2},\xi_{n-1},\;\xi_{n}\in V, \end{array}$$

in which *ξ*_1~*n*_ are the unit vectors with different directions.

$\overset{⟶}{OM}$ and $\overset{⟶}{ON}$ can be deduced as follows:

(7) $$\begin{array}{c} \overset{⟶}{OM}=m_{1}\cdot \xi_{1}+m_{2}\cdot \xi_{2}+m_{3}\cdot \xi_{3}+\cdots +m_{n-1}\cdot \xi_{n-1}+m_{n}\cdot \xi_{n},\\ \overset{⟶}{ON}=n_{1}\cdot \xi_{1}+n_{2}\cdot \xi_{2}+n_{3}\cdot \xi_{3}+\cdots +n_{n-1}\cdot \xi_{n-1}+n_{n}\cdot \xi_{n},\\ \overset{⟶}{MN}=\overset{⟶}{ON}-\overset{⟶}{OM},\\ \overset{⟶}{MN}=\left(n_{1}-m_{1}\right)\cdot \xi_{1}+\left(n_{2}-m_{2}\right)\cdot \xi_{2}+\cdots +\left(n_{n-1}-m_{n-1}\right)\cdot \xi_{n-1}+\left(n_{n}-m_{n}\right)\cdot \xi_{n},\\ \overset{⟶}{MN}=\left(n_{1},n_{2},n_{3},\cdots ,n_{n‐1},n_{n}\right)-\left(m_{1},m_{2},m_{3},\cdots ,m_{n‐1},m_{n}\right)=\left(n_{1}-m_{1},n_{2}-m_{2},n_{3}-m_{3},\cdots ,n_{n‐1}-m_{n‐1},n_{n}-m_{n}\right). \end{array}$$

For the vector that takes “*M*” as the starting point and point “*N*” as the ending point, $\overset{⟶}{MN}=\left(n_{1}-m_{1},n_{2}-m_{2},n_{3}-m_{3},\cdots ,n_{n-1}-m_{n-1},n_{n}-m_{n}\right)$ can be obtained. That is to say, the coordinate of $\overset{⟶}{MN}$ is the coordinate of “*N*” minus that of “*M*”.

Based on “attribute indexes” related to medicinal properties, we can analyze the “attribute indexes” of “Blank” and Chinese medicines to obtain corresponding blank values and attribute indicator values of Chinese medicines.

Then, in the *N*-dimensional space composed of attribute indexes, we record the ordered array of blank values as “blank spot” coordinates; at the same time, we take the ordered array of attribute indicator values of Chinese medicines as “medicinal properties spot” coordinates. In that way, the vector from “blank spot” to “medicinal properties point” is a vector that can represent medicinal properties of a Chinese medicine, whose coordinate is the coordinate of “medicinal properties spot” minus that of “blank spot”.

For example, when the medicinal properties of Chinese medicine “*H*” are characterized by attribute indexes *I*_1_, *I*_2_, and *I*_3_, the corresponding blank values *a*_0_, *b*_0_, and *c*_0_ can be obtained by analysis of attribute indexes *I*_1_, *I*_2_, and *I*_3_ of the blank group. In the same way, the attribute index values *a*_1_, *b*_1_, and *c*_1_ can also be obtained by analysis of attribute indexes *I*_1_, *I*_2_, and *I*_3_ of drug “*H*”. Then, in a three-dimensional space formed by attribute indexes *I*_1_, *I*_2_, and *I*_3_, blank values arranged in the order of (*I*_1_, *I*_2_, and *I*_3_) are taken as “blank spot” coordinates, which are recorded as (*a*_0_, *b*_0_, and *c*_0_). Moreover, the ordered array of attribute indicator values is taken as “medicinal properties spot” that is recorded as (*a*_1_, *b*_1_, and *c*_1_). Therefore, we can obtain that the vector from “blank point” to “medicinal point” is a vector that can represent medicinal properties of Chinese medicine “*H*”. The coordinate of the above vector can be expressed as follows:

**H** = (*a*_1_, *b*_1_, *c*_1_) − (*a*_0_, *b*_0_, *c*_0_) = (*a*_1_ − *a*_0_, *b*_1_ − *b*_0_, *c*_1_ − *c*_0_), in which **H** represents the medicinal properties of Chinese medicine “*H*”.

On the premise of same “attribute index”, different Chinese medicines have different attribute index values. Therefore, through the vector representation of medicinal properties, different vectors can represent the same medicinal properties of different traditional Chinese medicines. Further, according to the basic rationale of quantification of medicinal properties, the quantification of same medicinal properties of different Chinese medicines was carried out to obtain the quantitative value of medicinal properties that is represented by “*R*”, which can realize the quantitative comparison of same medicinal properties of different Chinese medicines. In the following part, we deduced the general theoretical formula of “*R*”.

### 2.3. Quantitative Value of Medicinal Properties “*R*”

The general theoretical formula of “*R*” was deduced based on basic rationale of quantification of medicinal properties and coordinate representation of vector.

Suppose that the two Chinese medicines with the same medicinal properties were drug “*A*” and drug “*B*”, respectively. There are “*n*” characterization indexes selected to characterize medicinal properties, which are recorded as (*I*_1_, *I*_2_, *I*_3_,…,*I*_*n*−1_, *I*_*n*_). Through analysis of each attribute index of blank, drug “*A*”, and drug “*B*”, the “medicinal properties spots” of drug “*A*”, drug “*B*”, and the “blank spot” are as follows:

- Blank spot: (*a*_1_, *a*_2_, *a*_3_, ⋯,*a*_*n*−1_, *a*_*n*_)^T^
- Medicinal properties spot of drug “*A*”: (*b*_1_, *b*_2_, *b*_3_, ⋯,*b*_*n*−1_, *b*_*n*_)^T^
- Medicinal properties spot of drug “*B*”: (*c*_1_, *c*_2_, *c*_3_, ⋯,*c*_*n*−1_, *c*_*n*_)^T^

*a*_1_~*a_n_*, *b*_1_~*b_n_*, and *c*_1_~*c_n_* are all different attribute index values that correspond to indexes *I*_1_ ~ I_*n*_, respectively.

Based on the vector representation of medicinal properties, we got the vector coordinates of drug properties of traditional Chinese medicines “*A*” and “*B*”, which are represented by “**α**” and “**β**”, respectively.

(8) $$\begin{array}{c} \alpha ={\left(x_{1},x_{2},x_{3},\cdots ,x_{n-1},x_{n}\right)}^{\text{T}}={\left(b_{1},b_{2},b_{3},\cdots ,b_{n-1},b_{n}\right)}^{\text{T}}-{\left(a_{1},a_{2},a_{3},\cdots ,a_{n-1},a_{n}\right)}^{\text{T}}={\left(b_{1}-a_{1},b_{2}-a_{2},b_{3}-a_{3},\cdots ,b_{n-1}-a_{n-1},b_{n}-a_{n}\right)}^{\text{T}},\\ \beta ={\left(y_{1},y_{2},y_{3},\cdots ,y_{n-1},y_{n}\right)}^{\text{T}}={\left(c_{1},c_{2},c_{3},\cdots ,c_{n-1},c_{n}\right)}^{\text{T}}-{\left(a_{1},a_{2},a_{3},\cdots ,a_{n-1},a_{n}\right)}^{\text{T}}={\left(c_{1}-a_{1},c_{2}-a_{2},c_{3}-a_{3},\cdots ,c_{n-1}-a_{n-1},c_{n}-a_{n}\right)}^{\text{T}}. \end{array}$$

For vectors “**α**” and “**β**”, through vector coordinate operation, we obtained the following information [23]:

1. Modulus of vectors **α** and **β** are ‖*α*‖ and ‖*β*‖

(9) $$\begin{array}{c} \left\|\alpha \right\|=\sqrt{\overset{n}{\underset{i=1}{\sum }}x_{i}^{2}}=\sqrt{x_{1}^{2}+x_{2}^{2}+\cdots +x_{n-1}^{2}+x_{n}^{2}},\\ \left\|\beta \right\|=\sqrt{\overset{n}{\underset{i=1}{\sum }}y_{i}^{2}}=\sqrt{y_{1}^{2}+y_{2}^{2}+\cdots +y_{n-1}^{2}+y_{n}^{2}}. \end{array}$$

Scalar product of vectors **α** and **β** is recorded as [*α*, *β*].

(10) $$\begin{array}{c} \left[\alpha ,\beta \right]=\overset{n}{\underset{i=1}{\sum }}x_{i}y_{i}=x_{1}y_{1}+x_{2}y_{2}+x_{3}y_{3}+\cdots +x_{n-1}y_{n-1}+x_{n}y_{n}. \end{array}$$

(2) Cosine value of angle *θ*

[**α**, **β**] = ‖*α*‖ · ‖*β*‖ · cos*θ*, in which *θ* is the angle between vectors **α** and **β**, so cos *θ* could be deduced that

(11) $$\begin{array}{c} \cos\theta =\frac{\left[\alpha ,\beta \right]}{\left\|\alpha \right\|\cdot \left\|\beta \right\|}. \end{array}$$

(3) Based on above formula, we got that

(12) $$\begin{array}{c} \cos\theta =\frac{\left[\alpha ,\beta \right]}{\left\|\alpha \right\|\cdot \left\|\beta \right\|}=\frac{\sum_{i=1}^{n}x_{i}y_{i}}{\sqrt{\sum_{i=1}^{n}x_{i}^{2}}\cdot \sqrt{\sum_{i=1}^{n}y_{i}^{2}}}=\frac{x_{1}y_{1}+x_{2}y_{2}+\cdots +x_{n-1}y_{n-1}+x_{n}y_{n}}{\sqrt{x_{1}^{2}+x_{2}^{2}+\cdots +x_{n-1}^{2}+x_{n}^{2}}\cdot \sqrt{y_{1}^{2}+y_{2}^{2}+\cdots +y_{n-1}^{2}+y_{n}^{2}}}. \end{array}$$

When Chinese medicine “*B*” was the reference drug, the codirectional ray where vector **β** is located was taken as EAMP. At the same time, ‖*β*‖ was taken as the metrical unit of medicinal properties. In addition, the vertical projection of vector **α** on EAMP is ‖**α**‖ · cos*θ*. According to the basic principles of quantification of medicinal properties, we obtained the quantitative value of drug properties of Chinese medicine “*A*” compared to drug “*B*”, with the quantitative value of drug properties represented by *R*_(*A*, *B*)_.

(13) $$\begin{array}{c} R_{\left(A,B\right)}=\frac{\left\|\alpha \right\|\cdot \cos\theta }{\left\|\beta \right\|}=\frac{\sum_{i=1}^{n}x_{i}y_{i}}{\sum_{i=1}^{n}y_{i}^{2}}=\frac{x_{1}y_{1}+x_{2}y_{2}+\cdots +x_{n-1}y_{n-1}+x_{n}y_{n}}{y_{1}^{2}+y_{2}^{2}+\cdots +y_{n-1}^{2}+y_{n}^{2}}. \end{array}$$

When Chinese medicines “*A*” and “*B*” were not specified as reference drugs, we took the codirectional ray where vector **γ** was located as EAMP, with the vector **γ** was the resultant vector of vector **α** and vector **β**. Moreover, ‖*γ*‖ was taken as the metrical unit of drug properties to quantify the drug properties of Chinese medicines “*A*” and “*B*”:

(14) $$\begin{array}{c} \gamma =\alpha +\beta ,\\ \gamma ={\left(z_{1},z_{2},z_{3},\cdots ,z_{n-1},z_{n}\right)}^{\text{T}}={\left(x_{1},x_{2},x_{3},\cdots ,x_{n-1},x_{n}\right)}^{\text{T}}+{\left(y_{1},y_{2},y_{3},\cdots ,y_{n-1},y_{n}\right)}^{\text{T}}={\left(x_{1}+y_{1},x_{2}+y_{2},x_{3}+y_{3},\cdots ,x_{n-1}+y_{n-1},x_{n}+y_{n}\right)}^{\text{T}},\\ \left\|\gamma \right\|=\sqrt{\overset{n}{\underset{i=1}{\sum }}z_{i}^{2}}=\sqrt{z_{1}^{2}+z_{2}^{2}+\cdots +z_{n-1}^{2}+z_{n}^{2}}. \end{array}$$

Suppose that the angle between **α** and **γ** is *θ*_1_, with the angle between **γ** and **β** is *θ*_2_:

(15) $$\begin{array}{c} \cos\theta_{1}=\frac{\left[\alpha ,\gamma \right]}{\left\|\alpha \right\|\cdot \left\|\beta \right\|}=\frac{\sum_{i=1}^{n}x_{i}z_{i}}{\sqrt{\sum_{i=1}^{n}x_{i}^{2}}\cdot \sqrt{\sum_{i=1}^{n}z_{i}^{2}}}=\frac{x_{1}z_{1}+x_{2}z_{2}+\cdots +x_{n-1}z_{n-1}+x_{n}z_{n}}{\sqrt{x_{1}^{2}+x_{2}^{2}+\cdots +x_{n-1}^{2}+x_{n}^{2}}\cdot \sqrt{z_{1}^{2}+z_{2}^{2}+\cdots +z_{n-1}^{2}+z_{n}^{2}}},\\ \cos\theta_{2}=\frac{\left[\beta ,\gamma \right]}{\left\|\beta \right\|\cdot \left\|\gamma \right\|}=\frac{\sum_{i=1}^{n}y_{i}z_{i}}{\sqrt{\sum_{i=1}^{n}y_{i}^{2}}\cdot \sqrt{\sum_{i=1}^{n}z_{i}^{2}}}=\frac{y_{1}z_{1}+y_{2}z_{2}+\cdots +y_{n-1}z_{n-1}+y_{n}z_{n}}{\sqrt{y_{1}^{2}+y_{2}^{2}+\cdots +y_{n-1}^{2}+y_{n}^{2}}\cdot \sqrt{z_{1}^{2}+z_{2}^{2}+\cdots +z_{n-1}^{2}+z_{n}^{2}}}. \end{array}$$

Similarly, the quantitative value of medicinal properties of drugs “*A*” and “*B*” represented by *R*_*A*_ and *R*_*B*_, respectively, can be deduced according to the basic rationale of quantification of medicinal properties.

(16) $$\begin{array}{c} R_{A}=\frac{\left\|\alpha \right\|\cdot \cos\theta_{1}}{\left\|\gamma \right\|}=\frac{\sum_{i=1}^{n}x_{i}z_{i}}{\sum_{i=1}^{n}z_{i}^{2}}=\frac{x_{1}z_{1}+x_{2}z_{2}+\cdots +x_{n-1}z_{n-1}+x_{n}z_{n}}{z_{1}^{2}+z_{2}^{2}+\cdots +z_{n-1}^{2}+z_{n}^{2}},\\ R_{B}=\frac{\left\|\beta \right\|\cdot \cos\theta_{2}}{\left\|\gamma \right\|}=\frac{\sum_{i=1}^{n}y_{i}z_{i}}{\sum_{i=1}^{n}z_{i}^{2}}=\frac{y_{1}z_{1}+y_{2}z_{2}+\cdots +y_{n-1}z_{n-1}+y_{n}z_{n}}{z_{1}^{2}+z_{2}^{2}+\cdots +z_{n-1}^{2}+z_{n}^{2}}. \end{array}$$

Based on the derivation of formulas *R*_(*A*, *B*)_, *R*_*A*_, and *R*_*B*_, we have summarized the general theoretical formula of quantitative value of drug properties that is denoted by “*R*”.

(17) $$\begin{array}{c} R=\frac{\left\|l\right\|\cdot \cos\theta }{\left\|L\right\|}=\frac{\sum_{i=1}^{n}j_{i}p_{i}}{\sum_{i=1}^{n}p_{i}^{2}}\left(n\geq 1\right). \end{array}$$

In above general theoretical formula, ‖*l*‖ is the modulus of vector **l** that denotes medicinal properties of test Chinese medicine. ‖*L*‖ is the length of metrical unit of drug properties, with vector **L** is a vector representing medicinal properties of reference Chinese medicine or a resultant vector that is synthesized by all vectors representing medicinal properties of test drugs. “*θ*” is the angle between **l** and **L**. “*j*_i_” is the *i*-th component of vector **l** coordinate. “*p*_*i*_” is the *i*-th component of vector **L** coordinate.

Combining mathematical vectors with linear algebra and Chinese medicinal properties, we proposed the QMP metric model and deduced the general theoretical formula of quantitative value of medicinal properties “*R*”. Theoretically based on QMP and “*R*” formula, we can analyze abstract medicinal properties such as the four natures and five flavors. In the following sections, to verify the feasibility of QMP, based on analysis of correlation between primary metabolites and “cold-hot” medicinal properties, we carried out quantitative analysis of “cold-hot” medicinal properties of traditional Chinese medicines.

## 3. Quantitative Analysis of “Cold-Hot” Medicinal Properties

### 3.1. Correlation Analysis between Primary Metabolites and “Hot-Cold” Medicinal Properties

According to theory of traditional Chinese medicines, “four natures” that contain cold, hot, warm, and cool can be mainly divided into two categories: “hot-warm” and “cold-cool”. On the other hand, relevant research shows that the “hot-warm” and “cold-cool” properties of traditional Chinese medicines have a certain correlation with their material basis [7, 8, 23]. From this perspective, through data mining and literature collation, we have obtained some primary metabolite information of Chinese medicines with different drug properties, including the total sugar (TS), polysaccharide (PS), monosaccharide (MS), total lipid (TL), total protein (TP), and amino acid (AA). Based on above indicators and relevant data (Table 1) [24–26], we analyzed the correlation between primary metabolites and “hot-cold” medicinal properties based on Fisher's analysis.

On the basis of above indicators TS, PS, MS, TL, TP, and AA, we established the identification model of medicine properties through Fisher's linear analysis for exploring correlation between primary metabolites and “cold-hot” medicinal properties.

As shown in Figure 3, blue represents “cold-cool” Chinese medicines; meanwhile, red represents “hot-warm” Chinese medicines. Based on Fisher's discriminant function: *Y* = 0.45 × AA − 0.05 × TP − 0.87 × TL − 0.41 × MS − 0.06 × PS − 0.19 × TS − 10.58, we could correctly distinguish the drug properties of traditional Chinese medicines in Table 1 and the correct rate of discrimination reaches up to 93.88%. When *Y* > 0, the corresponding traditional Chinese medicines are classified as “cold-cool” medicines; if *Y* < 0, it could be classified as “hot-warm” Chinese medicines. The Fisher's discriminant results are shown in Table 2, in which the medicinal properties of Gardeniae fructus, Eucommiae cortex, and Clematidis radix et rhizoma were misjudged.

Through the quantitative discriminant function composed of indexes TS, PS, MS, TL, TP, and AA, the “cold-hot” medicinal properties of 46 different traditional Chinese medicines can be correctly distinguished, except Gardeniae fructus, Eucommiae cortex, and Clematidis radix et rhizoma. In other words, there was a correlation between above six indicators and “cold-hot” medicinal properties to a certain extent. On the basis of quantitative discrimination, in the system composed of 46 kinds of traditional Chinese medicines except Gardeniae fructus, Eucommiae cortex, and Clematidis radix et rhizoma, TS, PS, MS, TL, TP, and AA could be used as characterization indexes of drug properties.

### 3.2. Quantification of “Cold-Cool” Medicinal Properties

On the premise of characterization indexes determined in Section 3.1, we carried out quantitative comparison of “cold-cool” drug properties of different traditional Chinese medicines. At the same time, we took the quantitative comparison of “cold-cool” drug properties of Phellodendri chinensis cortex, Coptidis rhizoma, and Menthae haplocalycis herba as an example to explain in detail.

#### 3.2.1. Vector Expression of “Cold-Cool” Drug Properties

Based on TS, PS, MS, TL, TP, and AA, we used different vectors to represent the “cold-cool” drug property of Phellodendri chinensis cortex, Coptidis rhizoma, and Menthae haplocalycis herba. Since the attribute of index is the content of a certain component in the traditional Chinese medicines, moreover, the control blank did not contain the component to be tested, and the blank values of TS, PS, MS, TL, TP, and AA are all “0”. As can be seen from Table 1, the Phellodendri chinensis cortex's indicator values of TS, PS, MS, TL, TP, and AA were 24.51, 2.79, 2.21, 3.41, 9.27, and 4.68, respectively. Then, in the six-dimensional space formed by attribute indexes TS, PS, MS, TL, TP, and AA, blank values arranged in order of (TS, PS, MS, TL, TP, AA) were taken as “blank spot” whose coordinates were recorded as (0, 0, 0, 0, 0, 0). The same ordered array of attribute indicator values was taken as “medicinal properties spot” whose coordinate is (24.51, 2.79, 2.21, 3.41, 9.27, 4.68). Therefore, vector **A** from “blank point” to “medicinal properties point” is a vector that can represent “cold-cool” drug properties of Phellodendri chinensis cortex.

(18) $$\begin{array}{c} A=\left(24.51,2.79,2.21,3.41,9.27,4.68\right)-\left(0,0,0,0,0,0\right)=\left(24.51,2.79,2.21,3.41,9.27,4.68\right). \end{array}$$

In the same way, vectors **B** and **C** represent “cold-cool” drug properties of Menthae haplocalycis herba and Coptidis rhizoma, respectively, as follows:

(19) $$\begin{array}{c} B=\left(18.55,0.60,4.54,2.81,3.27,6.56\right)-\left(0,0,0,0,0,0\right)=\left(18.55,0.60,4.54,2.81,3.27,6.56\right),\\ C=\left(38.59,2.54,6.96,0.73,5.77,11.26\right)-\left(0,0,0,0,0,0\right)=\left(38.59,2.54,6.96,0.73,5.77,11.26\right). \end{array}$$

In the light of vector coordinate of **A**, **B**, and **C**, we quantitatively compared “cold-cool” drug properties of Phellodendri chinensis cortex, Menthae haplocalycis herba, and Coptidis rhizoma through the calculation of “*R*”.

#### 3.2.2. Quantitative Comparison of “Cold-Cool” Drug Properties Based on “*R*”

When performing quantitative comparison of “cold-cool” drug properties, we used Coptis chinensis as a reference drug. At this time, the quantitative values of medicinal properties of Phellodendri chinensis cortex and Menthae haplocalycis herba compared to that of Coptidis rhizoma were recorded as *R*_(*A*, *C*)_ and *R*_(*B*, *C*)_, respectively. According to the general theoretical formula of quantitative value of drug properties, it can be calculated that

(20) $$\begin{array}{c} R_{\left(A,C\right)}=\frac{\sum_{i=1}^{n}j_{i}p_{i}}{\sum_{i=1}^{n}p_{i}^{2}}=\frac{\left(24.51\times 38.59\right)+\left(2.79\times 2.54\right)+\cdots +\left(9.27\times 5.77\right)+\left(4.68\times 11.26\right)}{38.59^{2}+2.54^{2}+\cdots +5.77^{2}+11.26^{2}}=0.63,\\ R_{\left(B,C\right)}=\frac{\sum_{i=1}^{n}j_{i}p_{i}}{\sum_{i=1}^{n}p_{i}^{2}}=\frac{\left(18.55\times 38.59\right)+\left(0.60\times 2.54\right)+\cdots +\left(3.27\times 5.77\right)+\left(6.56\times 11.26\right)}{38.59^{2}+2.54^{2}+\cdots +5.77^{2}+11.26^{2}}=0.49. \end{array}$$

Coptidis rhizoma is the reference drug, the quantitative value of whose medicinal properties “*R*_*C*_” can be obtained by self-comparison.

(21) $$\begin{array}{c} R_{C}=1.00. \end{array}$$

According to the calculation of quantitative value of drug properties, we obtained that *R*_*C*_ > *R*_(*B*, *C*)_ > *R*_(*A*, *C*)_. That is to say, in the comparison of “cold-cool” medicinal properties, Coptidis rhizoma is the most “cold-cool”, followed by Phellodendri chinensis cortex, with Menthae haplocalycis herba is the weakest. Above results are consistent with the cognition of traditional Chinese medicine theory to Coptidis rhizoma, Phellodendri chinensis cortex, and Menthae haplocalycis herba. The theory of TCM holds that Coptidis rhizoma, Scutellariae radix, and Phellodendri chinensis cortex are all “cold” in drug properties, with Coptis chinensis being the most especially [27], while Menthae haplocalycis herba is classified as “cool” in drug properties which is weaker than “cold” [28].

In addition, based on characterization indexes and relevant data, taking Coptis rhizoma as reference drug and through the calculation of formula “*R*”, the quantitative values of drug properties of other “cold-cool” traditional Chinese medicines have been also obtained. The results of quantitative values of “cold-cool” drug properties are shown in Table 3.

### 3.3. Quantification of “Hot-Warm” Medicinal Properties

Using the same method as quantifying “cold-cool” medicinal properties, we quantified “hot-warm” drug properties. When making quantitative comparisons, we took “Fuzi” as the reference drug to calculate. The results are shown in Table 4.

As shown in Table 4, for example, *R*_(Fuzi)_ = 1.00, *R*_(Curculiginis rhizoma)_ = 0.82, and *R*_(Aucklandiae radix)_ = 0.21. The results showed that “hot-warm” properties of Fuzi are greater than those of Curculiginis rhizoma and Aucklandiae radix, which are also in line with the theoretical perception of traditional Chinese medicine. In addition, The *R* values in Table 4 allowed us to compare the strength or weakness of “hot-warm” drug properties of different Chinese medicines mentioned above.

## 4. Analysis and Discussion

### 4.1. QMP and Quantification Value “*R*”

In this paper, we defined QMP as quantitative comparison of same medicinal properties of different Chinese medicines through quantification value of Chinese medicinal properties “*R*”. Why is a quantitative comparison of the same medicinal properties rather than different medicinal properties? Just as Newton's laws have their own conditions of applicability, many of theory may be deviated or even erroneous when they exceeded scope of application. QMP is achieved by means of quantification value of Chinese medicinal properties “R”. Theoretically, since “cold-cool” and “hot-warm” are opposing medicinal properties, their quantification value “*R*” should be a negative value. However, in practice, as medicinal property indicators are objective and specific, they have their corresponding indicator values rather than subjective assignments. Therefore, there are basically no cases where the metric is negative. In order to ensure that the metric model is accurate and reliable, we define QMP as quantitative comparison of same medicinal properties.

The quantification value “*R*” was derived based on vector representation of medicinal properties and rules of vector operations, which has a solid theoretical foundation in mathematics. It can be used to quantify and compare the strength or weakness of medicinal properties such as four natures, five flavors, and toxicity, which provide a scientific and objective method for quantitative comparison of medicinal properties. It is worth noting that QMP is actually a relative metric comparison. For example, in Section 3.2.2, we used Coptidis rhizoma as the reference drug for comparison of medicinal properties. In other words, when the reference drugs are different, we can obtain different “*R*” values. However, what “*R*” stands for is the same; it is a relative comparison of the strength or weakness of medicinal properties. Such that *R*_(*A*, *B*)_ and *R*_(*A*, *C*)_ represent the strength or weakness of medicinal properties of drug “*A*” in relation to that of drug “*B*” and drug “*C*”, respectively.

### 4.2. Discussion of Quantification for “Cold-Hot” Medicinal Properties

The “cold-hot” medicinal properties have characteristics of abstractness, ambiguity, subjectivity, etc. [5]. Researchers have carried out analyses from a number of perspectives with some success [7, 8, 24, 25]. Wang et al. studied on the differentiation of “cold-hot” medicinal properties based on primary metabolites [29]. Wang and Li constructed the identification model of “cold-hot” medicinal properties based on the GC-MS chromatogram of lipid components [30]. All of these are indicative of the relevance of primary metabolites to medicinal properties to some extent. In addition, a single main ingredient or active ingredient is not sufficient to characterize medicinal properties of TCMs. Therefore, we integrated information on primary metabolites for correlation analysis of medicinal properties.

For correlation analysis between primary metabolites and drug properties, we used Fisher's linear analysis. Firstly, primary metabolites TS, PS, MS, TL, TP, and AA were highly correlated, nonlinearity, and unclear statistical distribution, which may not make the data suitable for statistical testing. Secondly, Fisher's linear analysis can turn the dimension of high-dimensional data with nonlinearity, high correlation, and unclear statistical distribution characteristics into low-dimensional linear space for discriminant analysis, which is suitable for data analysis. Based on primary metabolites TS, PS, MS, TL, TP, and AA, the “cold-hot” medicinal properties can be well distinguished, which proves that above indicators are in connection with “cold-hot” medicinal properties of 46 Chinese medicines (except Gardeniae fructus, Eucommiae cortex and Clematidis radix et rhizoma). In this process, the correlation was based on discriminatory analysis of “cold-hot”, which is currently the commonly used and recognized method. In this context, we proposed the QMP and the quantification value “*R*”. It is expected to provide a reference for quantitative comparison of medicinal properties.

From point of view of material base of medicinal properties, based on correlation indicators of medicinal properties of primary metabolites TS, PS, MS, TL, TP, and AA, we completed a quantitative comparison of “cold-hot” medicinal properties of 46 Chinese medicines. A few results contradicted the perception of TCM theory, such as *R*_(Euodiae fructus)_ = 0.19 and *R*_(Corydalis rhizoma)_ = 1.01. Above *R* values indicated that Corydalis rhizoma is more “hot-warm” than Euodiae fructus, which was at odds with TCM theory. This may be due to errors in experimental measurements. However, most of the results of quantitative comparison are basically in line with the perception of TCM theory. It demonstrates that QMP has certain guiding significance for quantitative comparison of “cold-hot” medicinal properties. It is feasibility for “*R*” to achieve quantitative comparison of same drug properties of different Chinese medicines, which is helpful to promote process of modern Chinese medicine construction. In addition, the QMP has a highly flexible character. Based on the choice of indicators, it can be applied to many areas of analysis related to drug properties to quantify medicinal properties of TCMs or to integrate multiple fields of analysis related to medicinal properties to evaluate the strength or weakness of medicinal properties, which is in line with the trend in medicinal properties research [31]. However, the current research studies have obvious shortages. The quality of research methods used to analyze the relationship between material composition and CMP varies. Many studies use subjective analysis methods that rely too much on the personal experience of experts and lack credible standards. It is difficult to solve the complex nonlinear and diversity problems in CMP discrimination, prediction, and quantification by using difference analysis methods such as standard deviation and *t*-test.

## 5. Conclusion

In this paper, we present quantification of Chinese medicinal properties (QMP) and the quantification value of medicinal properties “*R*”. Through the calculation of quantitative value of drug properties “R”, we can realize the quantitative comparison of “cold-hot” medicinal properties of TCMs; that is to say, it is feasible for QMP to achieve the quantitative comparison of same drug properties of different Chinese medicines. In addition, QMP has certain guiding significance for the quantification of Chinese medicinal properties. It is beneficial to promote the process of modern Chinese medicine construction.

## Figures and Tables

**Figure 1:** Based rationale of quantitative analysis for medicinal properties with reference drug, in which EAMP is the evaluation axis of medicinal properties.

**Figure 2:** Based rationale of quantification of medicinal properties with no reference drug, in which EAMP is the evaluation axis of medicinal properties.

**Figure 3:** The diagram of Fisher's linear discriminant.

**Table 1:** Content results of relevant components in 49 traditional Chinese medicines (%).

	TCM	TS	PS	MS	TL	TP	AA
Cold-cool	Anemarrhenae rhizoma	27.83	6.42	5.25	1.21	4.02	6.73
	Gardeniae fructus	22.09	3.10	5.69	11.67	3.03	5.23
	Lophatherum herba	20.85	2.36	2.06	1.38	2.65	7.07
	Phellodendri chinensis cortex	24.51	2.79	2.21	3.41	9.27	4.68
	Coptidis rhizoma	38.59	2.54	6.96	0.73	5.77	11.26
	Fraxini cortex	31.55	0.70	1.97	0.61	1.42	1.55
	Lonicerae japonicae flos	16.17	4.33	10.38	2.09	8.73	9.34
	Isatidis folium	14.72	1.14	4.58	3.15	7.92	15.32
	Taraxaciherba	20.46	7.64	7.61	3.50	8.45	9.69
	Menthae haplocalycis herba	18.55	0.60	4.54	2.81	3.27	6.56
	Platycladi cacumen	12.93	1.48	5.79	4.06	2.77	5.65
	Bupleuri radix	23.22	0.84	2.74	3.23	3.67	4.75
	Plantaginis semen	18.51	1.09	2.14	5.02	1.73	10.40
	Kochiae fructus	29.91	2.40	2.72	8.18	14.21	14.39
	Puerariae lobatae radix	39.57	5.70	4.49	1.01	6.44	3.58
	Sargassum	9.46	2.06	3.27	0.30	0.24	3.91
	Dianthi herba	23.61	0.04	7.13	2.58	5.56	5.83
	Trichosanthis fructus	23.77	0.62	13.92	7.76	10.73	15.99
	Gentianae radix et rhizoma	39.42	1.54	7.86	2.20	1.52	8.14
	Aloe	9.18	0.17	16.41	0.20	3.44	1.96
	Trachelospermi caulis et folium	24.10	1.42	6.48	1.52	7.63	4.57
	Ecliptae herba	11.86	1.05	3.88	1.04	1.37	7.91
	Siegesbeckiae herba	13.05	1.30	7.03	6.33	4.19	4.88
	Arnebiae radix	13.36	0.43	3.25	1.86	3.43	3.28
Hot-warm	Fuzi	92.45	4.24	1.01	0.58	0.47	1.96
	Cinnamomi cortex	45.87	5.75	1.20	5.22	13.47	1.11
	Zingiberis rhizoma	65.03	4.14	11.07	4.72	15.32	5.40
	Euodiae fructus	17.28	2.54	11.35	7.31	13.99	5.32
	Alpiniae officinarum rhizoma	43.99	6.12	14.02	2.89	12.21	1.86
	Piperis fructus	55.48	5.53	2.91	6.61	0.47	8.60
	Piperis longi fructus	57.12	4.02	6.36	5.77	2.71	9.23
	Curculiginis rhizoma	74.68	4.29	12.43	1.53	63.08	10.87
	Eucommiae cortex	26.52	1.22	7.33	4.25	1.09	2.79
	Sinapis semen	20.12	0.75	2.00	25.05	21.19	24.26
	Pinelliae rhizoma	77.71	26.67	1.02	0.26	3.84	4.14
	Psoraleae fructus	19.73	0.24	9.11	15.06	39.86	23.35
	Atractylodis rhizoma	26.59	16.28	17.73	6.73	0.33	2.62
	Alpiniae katsumadai semen	52.48	3.17	2.98	8.70	0.84	6.20
	Citri reticulatae pericarpium	37.90	3.60	24.75	1.30	1.33	3.96
	Chuanxiong rhizoma	44.25	2.52	3.29	8.83	35.65	11.11
	Magnollae officinalis cortex	28.23	0.96	7.57	6.06	1.85	2.30
	Ephedrae herba	27.37	1.47	11.16	3.21	2.99	3.65
	Chaenomelis fructus	22.31	2.90	18.86	1.70	4.50	3.66
	Aucklandiae radix	17.92	33.22	18.90	5.57	2.98	4.05
	Notopthrygii rhizoma et radix	29.94	2.22	3.51	9.77	3.88	5.48
	Arisaematis rhizoma	93.82	12.95	2.24	0.48	0.64	4.31
	Clematidis radix et rhizoma	34.72	1.48	8.13	0.66	1.59	5.29
	Asari radix et rhizoma	71.77	5.09	5.67	1.31	4.40	4.97
	Corydalis rhizoma	93.25	11.50	3.96	0.51	1.01	8.34

**Table 2:** Fisher's discriminant results of 49 traditional Chinese medicines.

TCM	*Y*	Drug properties	Test classification
Anemarrhenae rhizoma	4.63	Cold-cool	Cold-cool
Gardeniae fructus	-4.03	Cold-cool	Hot-warm^∗∗^
Lophatherum herba	7.54	Cold-cool	Cold-cool
Phellodendri chinensis cortex	3.61	Cold-cool	Cold-cool
Coptidis rhizoma	4.51	Cold-cool	Cold-cool
Fraxini cortex	3.90	Cold-cool	Cold-cool
Lonicerae japonicae flos	5.05	Cold-cool	Cold-cool
Isatidis folium	9.68	Cold-cool	Cold-cool
Taraxaciherba	4.12	Cold-cool	Cold-cool
Menthae haplocalycis herba	5.56	Cold-cool	Cold-cool
Platycladi cacumen	4.59	Cold-cool	Cold-cool
Bupleuri radix	4.20	Cold-cool	Cold-cool
Plantaginis semen	6.40	Cold-cool	Cold-cool
Kochiae fructus	2.39	Cold-cool	Cold-cool
Puerariae lobatae radix	1.40	Cold-cool	Cold-cool
Sargassum	8.84	Cold-cool	Cold-cool
Dianthi herba	3.35	Cold-cool	Cold-cool
Trichosanthis fructus	0.35	Cold-cool	Cold-cool
Gentianae radix et rhizoma	1.55	Cold-cool	Cold-cool
Aloe	2.72	Cold-cool	Cold-cool
Trachelospermi caulis et folium	3.70	Cold-cool	Cold-cool
Ecliptae herba	9.31	Cold-cool	Cold-cool
Siegesbeckiae herba	1.68	Cold-cool	Cold-cool
Arnebiae radix	6.42	Cold-cool	Cold-cool
Fuzi	-7.14	Hot-warm	Hot-warm
Cinnamomi cortex	-3.57	Hot-warm	Hot-warm
Zingiberis rhizoma	-8.82	Hot-warm	Hot-warm
Euodiae fructus	-2.07	Hot-warm	Hot-warm
Alpiniae officinarum rhizoma	-6.02	Hot-warm	Hot-warm
Piperis fructus	-3.28	Hot-warm	Hot-warm
Piperis longi fructus	-3.99	Hot-warm	Hot-warm
Curculiginis rhizoma	-8.21	Hot-warm	Hot-warm
Eucommiae cortex	0.04	Hot-warm	Cold-cool^∗∗^
Sinapis semen	-5.96	Hot-warm	Hot-warm
Pinelliae rhizoma	-4.55	Hot-warm	Hot-warm
Psoraleae fructus	-1.33	Hot-warm	Hot-warm
Atractylodis rhizoma	-7.28	Hot-warm	Hot-warm
Alpiniae katsumadai semen	-5.53	Hot-warm	Hot-warm
Citri reticulatae pericarpium	-6.24	Hot-warm	Hot-warm
Chuanxiong rhizoma	-3.61	Hot-warm	Hot-warm
Magnollae officinalis cortex	-2.20	Hot-warm	Hot-warm
Ephedrae herba	-0.49	Hot-warm	Hot-warm
Chaenomelis fructus	-1.50	Hot-warm	Hot-warm
Aucklandiae radix	-5.56	Hot-warm	Hot-warm
Notopthrygii rhizoma et radix	-2.84	Hot-warm	Hot-warm
Arisaematis rhizoma	-7.26	Hot-warm	Hot-warm
Clematidis radix et rhizoma	2.39	Hot-warm	Cold-cool^∗∗^
Asari radix et rhizoma	-4.65	Hot-warm	Hot-warm
Corydalis rhizoma	-5.99	Hot-warm	Hot-warm

∗∗ represents a wrong judgment of drug properties.

**Table 3:** The results of quantitative values of “cold-cool” drug properties.

TCM	*R*	TCM	*R*
Anemarrhenae rhizoma	0.72	Kochiae fructus	0.84
Lophatherum herba	0.54	Puerariae lobatae radix	0.97
Phellodendri chinensis cortex	0.63	Sargassum	0.26
Coptidis rhizoma^∗∗^	1.00	Dianthi herba	0.62
Fraxini cortex	0.74	Trichosanthis fructus	0.74
Lonicerae japonicae flos	0.51	Gentianae radix et rhizoma	0.99
Isatidis folium	0.48	Aloe	0.30
Taraxaciherba	0.60	Trachelospermi caulis et folium	0.63
Menthae haplocalycis herba	0.49	Ecliptae herba	0.34
Platycladi cacumen	0.37	Siegesbeckiae herba	0.38
Bupleuri radix	0.58	Arnebiae radix	0.35
Plantaginis semen	0.51	—	—

Coptidis rhizoma^∗∗^ was taken as the reference drug.

**Table 4:** The results of quantitative values of “hot-warm” drug properties.

TCM	*R*	TCM	*R*
Fuzi^∗∗^	1.00	Alpiniae katsumadai semen	0.57
Cinnamomi cortex	0.50	Citri reticulatae pericarpium	0.41
Zingiberis rhizoma	0.71	Chuanxiong rhizoma	0.48
Euodiae fructus	0.19	Magnollae officinalis cortex	0.31
Alpiniae officinarum rhizoma	0.48	Ephedrae herba	0.30
Piperis fructus	0.60	Chaenomelis fructus	0.25
Piperis longi fructus	0.62	Aucklandiae radix	0.21
Curculiginis rhizoma	0.82	Notopthrygii rhizoma et radix	0.33
Sinapis semen	0.23	Arisaematis rhizoma	1.02
Pinelliae rhizoma	0.85	Asari radix et rhizoma	0.78
Psoraleae fructus	0.22	Corydalis rhizoma	1.01
Atractylodis rhizoma	0.30	—	—

## Data Availability

All the raw data could be accessed by contacting the corresponding author on reasonable request.
